The article "Axillary and internal mammary sentinel lymph node biopsy in breast cancer after neoadjuvant chemotherapy" was published in 2016. Journal: Oncotarget.

# Axillary and internal mammary sentinel lymph node biopsy in breast cancer after neoadjuvant chemotherapy

**DOI:** 10.18632/oncotarget.12615

**Published:** 2016-10-12

**Authors:** Xiao-Shan Cao, Hui-Juan Li, Bin-Bin Cong, Xiao Sun, Peng-Fei Qiu, Yan-Bing Liu, Chun-Jian Wang, Yong-Sheng Wang

**Affiliations:** ^1^ Breast Cancer Center, Shandong Cancer Hospital Affiliated to Shandong University, Jinan, Shandong, China; ^2^ Department of Medical Administration Division, Shandong Cancer Hospital affiliated to Shandong University, Jinan, Shandong, China; ^3^ School of Medicine and Life Sciences, University of Jinan and Shandong Academy of Medical Sciences, Jinan, Shandong, China

**Keywords:** breast cancer, neoadjuvant chemotherapy, sentinel lymph node biopsy, internal mammary, axilla

## Abstract

With the improvement of neoadjuvant chemotherapy (NAC), the proportion of pathological complete response (pCR) in the breast and axillary lymph node (ALN) is increasing. The evaluation of pCR does not include the status of internal mammary lymph node (IMLN). This study is to evaluate the roles of both axillary sentinel lymph node biopsy (ASLNB) and internal mammary sentinel lymph node biopsy (IM-SLNB) in breast cancer patients after NAC. There were 74 patients enrolled into this study. IM-SLNB was performed on patients with radioactive internal mammary sentinel lymph node (IM-SLN). Patients (*n* = 8) with cN0 and ycN0 received ASLNB, and axillary lymph node dissection (ALND) in cases of positive axillary sentinel lymph node (ASLN). Patients (*n* = 48) with cN+ but ycN0 received ASLNB and ALND. Patients (*n* = 18) with ycN+ received ALND without ASLNB. The visualization rate of IM-SLN was 56.8% (42/74). The success rate of IM-SLNB was 97.6% (41/42) and the metastasis rate of IM-SLN was 7.3% (3/41). The success rate of ASLNB was 100% (56/56). The false negative rate (FNR) of ASLNB was 17.2% (5/29). The FNR in patients with 1, 2 and ≥ 3ASLNs examined was 27.3% (3/11), 20.0% (2/10) and 0% (0/8) respectively. ASLNB could be performed on ycN0 after NAC, and ALND should be performed on initially ALN-positive patients. IM-SLNB should be considered after NAC, especially for patients with clinically positive axillary nodes before NAC, which might help make clear of the pathological nodal staging of both ALN and IMLN, improve the definition of nodal pCR, and guide the individual adjuvant regional and systemic therapy.

## INTRODUCTION

Neoadjuvant chemotherapy (NAC) has become the standard therapy for both locally advanced and early-stage breast cancer in recent years for the improvement breast-conserving surgery rate and the evaluation of treatment response *in vivo* [1, 2]. Pathological complete response (pCR) is an independent prognostic factor irrespective of breast cancer intrinsic subtypes after NAC [3], and the prognostic value is greatest in aggressive tumor subtypes [1]. Definition of pCR has changed from eradication of tumor in the breast alone (ypT0/is) to both the breast and lymph nodes (ypT0/is ypN0), which was better associated with improved event-free survival and overall survival and indicated the importance of the pathological status of axillary lymph node (ALN) [1, 2]. Axillary sentinel lymph node biopsy (ASLNB) has replaced axillary lymph node dissection (ALND) as the standard axillary nodal staging technique for patients with clinically node-negative (cN0) breast cancer [4]. The application of ASLNB for axillary staging after NAC on those who initially had node-positive (cN+) breast cancer is uncertain due to the high false-negative rate (FNR) reported in previous studies [5, 6]. Additionally, an increase of pCR rate did not predict improved survival rate absolutely, maybe it is related to that previous studies only evaluated the pathological status of ALN without internal mammary lymph node (IMLN) condition. This study is to evaluate the roles of both internal mammary sentinel lymph node biopsy (IM-SLNB) and ASLNB in breast cancer patients after NAC.

## RESULTS

### Patient characteristics

A total of 74 patients with T0-4, N1-3, and M0 breast cancer were enrolled into this study, and the median age was 48.5 years (range, 27 to 68 years). All of the demographic and clinic-pathologic characteristics were listed in Table 1.

**Table 1:** Clinical and pathological characteristics of the enrolled patients

Characteristic	No.	%
Subgroup	74	
cN0→ycN0	8	10.8
cN+→ycN0	48	64.9
cN+→ycN+	18	24.3
Clinical tumor size before chemotherapy (cm)		
≤ 2	10	13.5
> 2 and ≤ 5	44	59.5
> 5	20	27.0
Clinical node stage before chemotherapy		
cN0	8	10.8
cN1	34	45.9
cN2-3	32	43.3
Subtype		
Luminal A	11	14.9
Luminal B/ HER-2-	18	24.3
Luminal B/ HER-2+	13	17.6
HER-2 +	14	18.9
Triple negative	18	24.3
Pathological node stage		
ypN0	26	35.1
ypN1	22	29.8
ypN2-3	26	35.1

### IM-SLNB

The visualization rate of internal mammary sentinel lymph nodes (IM-SLNs) was 56.8% (42/74). The median age of these 42 patients was 50 years (range, 32-68 years). The clinical and pathological characteristics of the patients with and without IM-SLN visualization were listed in Table 2. Patients body mass index, tumor location, and axillary nodal stage did not affect the IM-SLN visualization rate (all *P* > 0.05). The clinical tumor size before NAC was negatively correlated with the IM-SLN visualization rate (*P* = 0.004, Table 2).

**Table 2:** Clinical and pathological characteristics of the patients with and without IM-SLN imaging

Characteristic	Patients of IM-SLN visualized *(n* = 42)	Patients of IM-SLN not visualized (*n* = 32)	*P* value
Subgroup			0.864
cN0→ycN0	4	4	
cN+→ycN0	27	21	
cN+→ycN+	11	7	
Clinical tumor size before NAC (cm)			0.004
≤ 2	7	3	
> 2 and ≤ 5	30	14	
>5	5	15	
Clinical node stage before NAC			0.677
cN0	4	4	
cN1	18	16	
cN2-3	20	12	
Tumor Location			0.112
Outer	31	16	
Inner	4	7	
Center	7	9	
Pathological node stage			0.518
ypN0	13	13	
ypN1	12	10	
ypN2-3	17	9	
BMI			0.260
18.5~24.99	21	20	
25~28	11	9	
> 28	10	3	

Abbreviations: NAC neoadjuvant chemotherapy; BMI body-mass-index.

The success rate of IM-SLNB was 97.6% (41/42). The median number of IM-SLNs was 2 (total 67, range 1-4). The site of IM-SLNs concentrated in the second (48.8%, 20/41) and third (58.5%, 24/41) intercostal space, and 24.4% (10/41) IM-SLNs both located in the second and third intercostal space. The median time-consuming of IM-SLNB was 10min (range 5–30 min).

The IM-SLN positive rate was 7.3% (3/41), and all of them combined with positive ALNs. The positive IM-SLN located in the second intercostal space in two patients, and the third intercostal space in one patient.

Only two patients had intraoperative surgical complications. One had injury to pleura which was repaired intraoperatively without pneumothorax on postoperative chest radiography. Internal mammary artery was injured in the other and was resolved intraoperatively without postoperative bleeding.

### ASLNB

There were eight patients with clinical node-negative before (cN0) and after (ycN0) NAC. The success rate of ASLNB was 100% (8/8), and the median number of axillary sentinel lymph nodes (ASLNs) was 3 (total 26, range 2–6). Two patients (2/8) with positive ASLNs received ALND.

There were 48 patients with cN+ to ycN0. The success rate of ASLNB was 100% (48/48). The median number of ASLNs was 2 (total 106, range 1–6). The accuracy rate of ASLNB was 89.6% (43/48). ASLNB was false-negative in 17.2% (5/29) of these patients. The FNR in patients with 1, 2 and ≥ 3 ASLNs biopsied was 27.3% (3 of 11), 20.0% (2 of 10) and 0% (0/8), respectively. There were 29 patients with cN1 disease, and the FNR of ASLNB was 20.0% (4/20). The FNR in patients with 1, 2 and ≥ 3 ASLNs examined was 33.3% (2/6), 33.3% (2/6) and 0% (0/8), respectively. There were 19 patients with cN2-3 disease, and the FNR of ASLNB was 11.1% (1/9). The FNR in patients with 1 and 2 ASLNs examined was 20% (1/5) and 0% (0/4).

There were 18 patients with clinical node-positive after NAC (ycN+). All of these patients except one (94.4%, 17/18) were found to have residual positive ALN.

### Outcome associated with pCR

28.4% (21/74) patients had eradication of tumors in breast, and 30.3% (20/66) patients had eradication of tumors in ALN. 17.6% (13/74) patients had eradication of tumors in both breast and lymph nodes, so the pCR rate was 17.6%. Seven of them were triple negative, and six of them were human epidermal growth factor (HER-2) positive (three of them received trastuzumab therapy before surgery).

## DISCUSSION

The pathology status of ALN is one of the strongest prognostic factors for patients with breast cancer and guides adjuvant loco-regional and systemic therapy decisions [7]. ASLNB after chemotherapy is as accurate for axilla staging as ASLNB prior to chemotherapy in cN0 patients, and ASLNB after chemotherapy results in fewer positive ASLNs and ALND [8]. The 2014 Sentinel Lymph Node Biopsy American Society of Clinical Oncology Clinical Practice Guideline [9] and 2016 National Comprehensive Cancer Network (NCCN) Breast Cancer Clinical Practice Guidelines [10] recommended that ASLNB might be offered before or after NAC, but the procedure seemed less accurate after NAC. The 2015 St. Gallen International Expert Consensus recommended that sentinel node biopsy was feasible and accurate after NAC and allowed precise assessment of pCR [11]. At present, the application of ASLNB for women who initially had cN+ converting to ycN0 was uncertain due to its relatively high FNR (> 10%) [5, 6].

This study showed that ASLNs were detected in all patients, whereas the overall FNR of ASLNB was 17.2% (5/29) for patients who converted from cN+ to ycN0 after NAC. Several studies have indicated that the FNR could be improved by marking the biopsy-proven positive nodes, using dual tracer, and removing more than two ASLNs [10, 12, 13]. Full course of NAC with anthracycline- and taxane-based regimens were performed in our study, and dual tracers (combination blue dye and ^99m^Tc-labeled sulfur colloid [^99m^Tc-SC]) were used for ASLNB with the median ASLNs number as two. The FNRs were 27.3 % (ACOSOGZ1071 31.5% [6], SENTINA 24.3% [7], SNFNAC 18.2% [13]) and 20.0% (ACOSOGZ1071 21.2% [6], SENTINA 18.5% [7]) with one to two ASLNs removed, respectively. The FNR was reduced to 0% with three or more ASLNs removed (ACOSOGZ1071 9.1% [6], SENTINA 4.9% [7]), which could be acceptable for clinical trials (< 10%). The SNFNAC study [13] indicated that a low ASLNB FNR (8.4%) could be achieved with mandatory use of immunohistochemistry (IHC) in patients with biopsy-proven node-positive after NAC. In this study, 94.4% patients with ycN+ were found residual node-positive disease, indicating that ASLNB should not be performed in patients with abnormal ALN revealed by ultrasound. ACOSOGZ1071 trial [14] showed that patients with normal ultrasound underwent ASLNB (with ≥ 2 ASLNs) would potentially reduce the FNR. With the modified technique above reducing FNR, patients with lower axilla tumor burden might avoid ALND after NAC. Kim et al [15] pointed out that ASLNB in initial cN+ to ycN0 patients might help identify axillary down staging and avoid ALND and its morbidity. It should be validated by large prospective randomized clinical trials to evaluate outcomes with long time follow-up. In those patients with positive ASLNs after NAC, whether axillary radiation could replace ALND is being evaluated in the Alliance A11202 clinical trial [14]. Individual management of axilla needs further studies.

The definition of pCR (ypT0/is ypN0) just included the evaluation of ALN [2]. As IMLN metastasis has similar prognostic importance as that of ALN [16–18], the lymphatic metastasis and down-stage should involve not only ALN but also IMLN. It is necessary to perform IM-SLNB after NAC to make clear of the whole nodal staging as there were still 7.3% of patients with IM-SLNs metastases after NAC.

High risk factors of IMLNs metastases including: ≥ 4 positive ALNs, medial tumor and positive ALNs, T3 tumor and younger than 35-year-old, T2 tumor and positive ALNs, and T2 tumor and medial tumor. The incidences of IMLNs metastasis for these patients were more than 20% [19]. The IMLN metastasis rate was higher in patients with ALN-positive than those with ALN-negative [16–18, 20]. Most patients received NAC were in the advanced stage with high risk of IMLN metastasis, so it was necessary to make clear the pathology status of IMLN in these patients. The 2016 NCCN Breast Cancer Clinical Practice Guidelines [10] recommended that adjuvant radiation therapy post-lumpectomy or post-mastectomy was based on pre-chemotherapy tumor characteristics as that radiation therapy to chest wall plus infraclavicaular region, supraclavicular area, internal mammary nodes, and any part of the axillary bed at risk to patients with ≥ 4 positive axillary nodes after surgery (category 1), which was category 2B in the 2015 NCCN guideline. It means that more and more attention was paid to the regional control of IMLN. However, some patients with IMLN-negative would receive over-treatment, and those with IMLN-positive but ALN-negative would receive under-treatment. Therefore, pathological status of IMLN is superior to high risk factors for the guidance of adjuvant therapy, and IM-SLNB could help to identify the metastasis in IM-SLN. For patients without NAC, internal mammary radiotherapy could be avoided in those with negative IM-SLN [17, 21], while it is still in dispute and needs our further exploration in those patients with negative IM-SLN after NAC.

The low visualization rate of IM-SLN is the restriction for both clinical study and daily practice of IM-SLNB [17, 18]. The modify radiotracer injection technique [18] (high volume, intraparenchyma, ultrasonographic guidance) broke through the bottle-neck of the low internal mammary visualization rate with traditional injection (71.1% vs. 15.5%, *P* < 0.001) in patients without NAC, and the radioactive IM-SLN could be detected in more than half of the patients (56.8%, 42/74) in this study after NAC. In 42 patients with radioactive IM-SLN, 41 patients (97.6%) received IM-SLNB successfully, and two patients (4.8%) occurred complications, which were in the acceptable range. IM-SLNB is safe and feasible [17, 18, 22], and should be recognized and taken into practice. The definition of pCR would not be complete without including the pathology status of IMLN.

ASLNB could apply to patients with both cN0 and ycN0. ALND should be performed on patients with cN+ due to the relatively high FNR at present. With dual tracers and ≥ 3 ASLNs biopsied, the FNR could decrease to be less than 10% in patients with cN+ converting to ycN0. For these patients, whether ASLNB could replace ALND needs to be validated by large prospective randomized clinical trials to evaluate outcomes with long time follow-up, ALND is still the standard method to be performed. IM-SLNB should be considered after NAC, especially for patients with clinically positive axillary nodes before NAC, which might help to make clear of the pathological nodal staging including both ALN and IMLN, improve the definition of nodal pCR, and guide the individual adjuvant regional and systemic therapy.

## MATERIALS AND METHODS

### Patients

In the study, 74 female patients who had histologically proven clinical stage T1-T4, N0-N3, M0 primary invasive breast cancer treated at our breast cancer center between January 2012 and October 2015 were enrolled. Full course of NAC with anthracycline- and taxane-based regimens were performed before surgery. HER-2 positive were identified in 27 patients, and six of them received anti-HER-2 targeted therapy (trastuzumab) before surgery. Patients with inflammatory breast cancer and with a history of prior ipsilateral axillary surgery or radiotherapy, prior ASLNB, or excisional lymph node biopsy for pathology confirmation of axillary pathological status were excluded. The study was approved by the Shandong Cancer Hospital Affiliated to Shandong University Ethics Committee (No. SDTHEC20130324), informed consent was obtained from the patients and all procedures were in accordance with the ethical standards of the responsible institutional committee on human experimentation and with the Helsinki Declaration.

### Study design and procedure

For all patients, 18.5-–37 MBq of ^99m^Tc-SC in 1.0–1.2 ml volume was injected intraparenchymally at the 6 and 12 o'clock positions 2.0-3.0 cm away from the nipple under ultrasonographic guidance 3-18 h before surgery. Subsequently, lymphoscintigraphy was performed 0.5-1.0 h before surgery (Figure 1). Additionally, blue dye (methylene blue) was injected subcutaneously into the breast 10 min before surgery.

**Figure 1:** SPECT(1a) and SPECT/CT(1b) image before operation A: radioactive IM-SLN, B and C: injection point, D:radioactive ASLN, ANT: anterior imaging, LL: left lateral imaging

IM-SLNB [21, 23] was performed on all patients with radioactive IMLN detected by preoperative lymphoscintigraphy and intraoperative gamma-probe (Figure 2).

**Figure 2:** Intraoperative IM-SLNB (**A**) and (**B**): IM-SLNB performed after lumpectomy with intraoperative gamma probe guided; (**C**) and (**D**): IM-SLNB performed after total mastectomy.

Women with clinically (palpation and ultrasound) node-negative disease before (cN0) and after (ycN0) NAC underwent ASLNB and received no further axillary surgery if they had a negative sentinel lymph node (ypN0sn). The ASLN was examined intraoperatively with imprint cytology (touch preparation) and frozen section [24]. Those had positive axilla nodes (fine needle aspiration) before NAC (cN+) and converted to clinically (palpation and ultrasound) node-negative disease after NAC (ycN0) underwent ASLNB following ALND. Patients with positive axillary node both before and after NAC received ALND without ASLNB (Figure 3). Radioactive and/or blue stained lymph nodes were identified as ASLNs, and palpably abnormal lymph nodes were also considered as ASLNs [6].

**Figure 3:** Study design program

### Pathology evaluation

All the sentinel lymph nodes were incised into two sections, embedded in paraffin and Hematoxylin &Eosin stain was used. Sentinel lymph node with metastases of any size were considered positive, including ypN1mi (> 0.2 to 2 mm) and ypN0(i) (≤ 0.2 mm).

### Statistical analysis

The data were analyzed with the SPSS 17.0 software package. Two-sample *t* test was used for continuous variables, and Pearson χ² test or Fisher exact test was used for categorical variables. All tests were two-sided, and *P* < 0.05 was considered statistically significant.
